# Detection of Pine Cones in Natural Environment Using Improved YOLOv4 Deep Learning Algorithm

**DOI:** 10.1155/2021/5601414

**Published:** 2021-12-16

**Authors:** Ze Luo, Yizhuo Zhang, Keqi Wang, Liping Sun

**Affiliations:** ^1^College of Mechanical and Electrical Engineering, Northeast Forestry University, Harbin 150040, China; ^2^School of Electrical Information Engineering, Hunan Institute of Technology, Hengyang 421010, China

## Abstract

Achieving the rapid and accurate detection of pine cones in the natural environment is essential for yield estimation and automatic picking. However, the complex background and tiny target pose a significant challenge to pine cone detection. This paper proposes a pine cone detection method using the improved You Only Look Once (YOLO) version 4 algorithm to overcome these challenges. First, the original pine cone image data come from a natural pine forest. Crawler technology is utilized to collect more pine cone images from the Internet to expand the data set. Second, the densely connected convolution network (DenseNet) structure is introduced in YOLOv4 to improve feature reuse and network performance. In addition, the backbone network is pruned to reduce the computational complexity and keep the output dimension unchanged. Finally, for the problem of feature fusion at different scales, an improved neck network is designed using the scale-equalizing pyramid convolution (SEPC). The experimental results show that the improved YOLOv4 model is better than the original YOLOv4 network; the average values of precision, recall, and AP reach 96.1%, 90.1%, and 95.8%; the calculation amount of the model is reduced by 21.2%; the detection speed is fast enough to meet the real-time requirements. This research could serve as a technical reference for estimating yields and automating the picking of pine cones.

## 1. Introduction

Pine nuts are commonly used in traditional recipes in many countries since they have rich flavor and nutritional benefits [1]. Pine nuts come from pine cones, and farmers are still the main force of pine cone picking. During the pine cone harvest, workers need to knock the pine cones off the tree and collect them on the ground. This work is time-consuming and high-risk. At the same time, workers who lack knowledge and experience make unnecessary mistakes, bringing more uncertainties to production. With the development of information technology, autonomous robots have become an essential means for yield estimation and automatic harvesting and have been widely used in the agriculture and forestry domains [2–4]. As part of the robot system, machine vision recognition might be one of the crucial technologies [5]. Therefore, designing a machine vision system for detecting pine cones on trees and the ground in a natural environment can provide technical support for pine cone yield estimation and the entire automatic picking process, which is of great significance.

Machine vision technology has been primarily used in agriculture and forestry for a long time, and many methods have been developed to detect fruits based on images. Lu et al. [6] proposed a layered contour analysis method based on shape features to detect immature citrus. Malik et al. [7] developed algorithms to detect ripe tomatoes according to color space and watershed. Li et al. [8] proposed a method of identifying green apples. This method combines texture features, shape features, and color features and is then segmented using support vector machines. However, the previously mentioned methods rely on shallow feature extraction and cannot solve the problems caused by overlap and occlusion. In addition, due to complex backgrounds and variable lighting, these methods cannot achieve desirable results in actual production environments [9].

Deep learning has rapidly evolved in recent years. Due to its ability to extract high-dimensional features from massive information, deep learning technology is more accurate than traditional methods [10]. Based on deep learning technology, researchers have developed a series of fruit detection methods [11]. Tu et al. [12] proposed a method for passion fruit detection based on multiple scale faster region-based convolutional neural networks, with the F1 score of 0.909, which effectively improves small passion fruit detection. Kirk et al. [13] combined biologically inspired features with one-stage deep learning networks to detect strawberries and achieved a detection speed of 30 fps on 1920 × 1080 pixels images. Liang et al. [14] considered the impact of light conditions on fruit recognition. They proposed combining the You Only Look Once (YOLO) network and U-Net, which can effectively detect litchi in the night environment. Although the previously mentioned methods have achieved desirable results in practical application, pine cone detection still faces many challenges. First, sufficient data is a necessary condition for using deep learning techniques [15]. However, the complex pine forest environment makes it challenging to collect pine cone images, and there is no public dataset of pine cones available online. On the other hand, the detection environment of pine cones is more complicated than other fruits, which leads to unsatisfactory results of existing algorithms. Moreover, the pine cone detection task has unique and complex features and requires high speed and accuracy. Since the tiny target is smaller, the algorithm will be less accurate in predicting location information than the larger target. In actual production, detection speed is one of the most critical factors, and pine cone detection requires high real-time performance. Because of the previously mentioned reasons, applying deep learning technology in pine cone detection is still a problem to be solved urgently.

As a current excellent one-stage detection algorithm, the YOLO [16–18] series algorithm is widely used in various target detection tasks [19–21]. The YOLO algorithm directly uses the regression to detect objects, which effectively improves the detection speed. In addition, due to the excellent network structure design, the YOLO algorithm also has a higher detection accuracy. In previous research, we combined boundary equilibrium generative adversarial networks and YOLOv3 to detect pine cones and achieved certain results [22]. However, this method is only for pine cones on the ground, and its accuracy and speed need to be further improved. Compared with the YOLOv3 algorithm, the YOLOv4 [23] algorithm owns a more balanced speed and accuracy and can be better applied to the actual working environment. However, for the pine cone detection task, the backbone and neck networks of YOLOv4 have room for further improvement. Therefore, this paper designs a new pine cone detection algorithm based on YOLOv4. Its main contributions are as follows. First, we manually collected more images of pine cones based on the previous work. All images were collected in a natural pine forest. At the same time, we used crawler technology to obtain images from the Internet to expand the dataset. Second, we introduced the densely connected convolution network (DenseNet) structure in the YOLOv4 model, which improves the detection performance of the model through feature reuse. Then, we pruned the backbone network to reduce the computational complexity and keep the output dimension unchanged. Finally, to improve the performance of small target detection, we used the idea of scale-equalizing pyramid convolution (SEPC) for reference and designed an improved neck network to achieve feature fusion between different scales.

The rest of this article is organized as follows.  Section 2 introduces the data set; Section 3 introduces the YOLOv4 model and related improvements methods; Section 4 introduces the experimental configuration, comparative experiment results, and discussion; Section 5 introduces the conclusions and prospects of this article.

## 2. Dataset and Data Augmentation

### 2.1. Dataset

In this research, we first manually collected 961 images of pine cones from a forest farm in Jiamusi City, Heilongjiang Province, China from 2019 to 2020. Then, to simulate the complex detection background, we developed a web crawler program to download pine cone images from the Internet. The primary sources of downloaded images are Google and free gallery websites. After manual screening, 450 images are obtained. Finally, we got a pine cone dataset containing 1411 images and divided it into training and validation set according to 8 : 2.

The dataset of this research had the following characteristics. For target selection, the images collected in the dataset include pine cones on the ground, pine cones on trees, mature pine cones, and immature pine cones. Therefore, the method proposed in this research can provide a technical reference for the complete pine cone harvesting process. In addition, we considered the impact of different light intensities: the images were collected on sunny and cloudy days, and the collection time included 8 am, 1 pm, and 3 pm. Moreover, the web crawler technology enriched the detection background of pine cone images and ensured the detection method was more robust.  Figure 1 illustrates different pine cone images from the dataset.

### 2.2. Data Augmentation

A data augmentation strategy can increase the richness of the experimental data and simulate the complex scenes of object detection more effectively, thereby improving the model's performance [24]. In this research, in addition to the five standard data augmentation methods (flipping, rotation, scaling, clipping, and brightness adjustment), Mosaic was used to augment the data. Mosaic is a further extension of the CutMix [25] data augmentation algorithm. It combines four training images into one in specific ratios, which can improve the model's recognition ability under complex backgrounds and the accuracy of detecting small targets.  Figure 2 shows the effect of data augmentation.

## 3. Methods

### 3.1. YOLOv4

YOLOv4 is a high-precision and real-time one-stage target detection algorithm proposed by Alexey in April 2020, which has been recognized by the original author of the YOLO series. As illustrated in Figure 3, the YOLOv4 model mainly consists of three components: backbone network, neck network, and prediction network.

The backbone network of YOLOv4 is named CSPDarkNet53, which combines the advantages of DarkNet53 [18] and Cross-Stage Partial Network (CSPNet) [26]. In YOLOv4, the CSPDarknet53 consists of 5 CSP modules, and each CSP module contains several residual layers. By using the cross-stage hierarchy, the CSP module divides the feature mapping of the foundation layers into two parts. By integrating gradient change into the feature map from beginning to end, the amount of calculation can be reduced, and accuracy can be ensured. Therefore, using the CSP module instead of the ordinary convolution layer can solve the gradient disappearance problem and overfitting problem caused by the dense network and make the model more lightweight and accurate.

The neck network is a series of feature aggregation layers that combine image features. YOLOv4 combines Spatial Pyramid Pooling (SPP) [27] and PAN [28] to form the neck network. In the SPP structure, the input from backbone undergoes four different max-pooling operations to further extract and fuse features. The PAN fuses the feature layers input from the SPP and the backbone network and sends them to the prediction network for detection. As shown in Figure 4, unlike the feature pyramid network (FPN) in YOLOv3, YOLOv4 builds a bottom-up feature transfer path by adding two PAN structures, which improves the transmission of low-level features and enhances the detection of targets of different scales.

### 3.2. Improved Methods

The main improvements presented in this paper based on YOLOv4 are as follows: introduce the DenseNet structure, prune the backbone network, and design an improved neck network.

#### 3.2.1. Backbone Network

The CSP module in the YOLOv4 backbone network uses ResNet [29] structure to solve the problem of overfitting and gradient disappearance. But, for the pine cone detection task, most of the targets that need to be detected are tiny targets, and the feature semantic information extraction by shallow networks is more critical. Similar to the ResNet structure, the DenseNet [30] structure optimizes the network by linking the front and rear layers. The difference is that the ResNet structure only establishes links between part of the front and rear layers, while DenseNet structure establishes links between all the front and rear layers. Therefore, the DenseNet can better transfer the feature semantic information to the depths of the network. The principle of DenseNet is shown in (1). Assuming the input is *X*_0_, *i*  represents the *i* th layer; each layer implements a nonlinear transformation *H*_*i*_(.) and then the output of *i* th layer as *X*_*i*_.

(1) $$\begin{array}{c} X_{i}=H_{i}\left(\left[X_{0},X_{1},\ldots ,X_{i-1}\right]\right). \end{array}$$

The original YOLOv4 model has 5 CSP modules. Replacing them with the CSPDenseNet module can further strengthen the transmission of shallow feature information in the network. However, when the structure composition is the same, the CSPDenseNet module has more parameters than the CSP module. Using the CSPDenseNet module to replace all CSP modules will significantly increase the amount of calculation, reduce the detection speed of the model, and cannot guarantee to improve the detection accuracy. The 3rd, 4th, and 5th CSP modules are located at a deeper level of the network. Replacing them with CSPDenseNet modules can better solve the problem of gradient disappearance and achieve the balance between performance and speed. Therefore, this paper used the CSPDenseNet module to replace the 3rd, 4th, and 5th CSP modules. As shown in Figure 5, the CSPDenseNet module divides the input into two parts, one part is calculated by the dense block, and the other part is connected through a cross-stage hierarchy. The dense block consists of several dense layers, and each dense layer contains two convolutional operations, 1 × 1 and 3 × 3. The 1 × 1 convolution operation is used to adjust the input dimension and reduce computational complexity, and the 3 × 3 convolution operation is used to enhance feature extraction. Then, any two dense layers are connected by a shortcut link.

In the original YOLOv4, the CSP module uses Mish as the activation function, and other modules use Leaky-ReLU as the activation function. Mish nonlinearity improves the accuracy, but in the embedded environment, its computing cost is more expensive than the Leaky-ReLU. Compared with Mish, SiLU [31] has similar performance and lower computational cost. In order to reduce the computational complexity, the Mish activation function in the model has been changed to SiLU, and the Leaky-ReLU remains unchanged.

The number of filters in the dense layer will affect the performance of the network. Too many filters will result in complicated calculations, and too few filters will result in insufficient feature extraction. Referring to the original residual block in YOLOv4, we set the number of filters for 1  × 1 convolution to 64, 128, and 256 and the number of filters for 3 × 3 convolution to 32, 64, and 128. In addition, the five original CSP modules contain 1, 2, 8, 8, and 4 residual layers, respectively. To reduce the computational complexity and keep the output dimension unchanged, we pruned the network structure by setting the number of dense layers in each CSPDenseNet structure to 4.  Table 1 shows the original backbone structure and the improved backbone network structure.

#### 3.2.2. Neck Network

Neck network is a key link in the target detection framework. It reprocesses the features extracted by backbone to generate a feature pyramid, which will enhance the model's detection of objects at different scales. Before the emergence of path aggregation network (PAN), feature aggregation in the target detection framework was generally implemented using FPN. FPN only has a top-down feature transfer path, and PAN has added a bottom-up feature transfer path to enhance the effect of feature fusion.

Although PAN enhances the fusion of features, it does not consider the intrinsic properties of the feature pyramid and can be further improved. Wang et al. [32] proposed the SEPC to explore the interaction between different scales of the feature pyramid. The SPEC is a 3D convolution composed of N 2D convolutions, which include scale and spatial dimensions. The difference between SPEC, FPN, and PAN is shown in Figure 6. For each feature fusion calculation, SEPC adds shallower and deeper features, which is equivalent to combining the advantages of FPN and PAN. When multiple SEPC modules are combined, its advantages in spatial dimensions will be more obvious.

The calculation process of SEPC is shown in (2): *y* is the output, *X* is the input feature map of different scales, *ω*_1_, *ω*_0_, and *ω*_−1_ are three independent 2D convolutional kernels, and *S*_*n*_ represents the stride of the convolution kernel  *n*. When calculating the top level of the feature pyramid, the first item is unnecessary, and when calculating the bottom level, the last item is unnecessary.

(2) $$\begin{array}{c} y^{l}=\omega_{1}*S_{0.5}X^{l+1}+\omega_{0}*S_{1}X^{l}+\omega_{-1}*S_{2}X^{l-1}. \end{array}$$

When the stride of the convolution kernel *n* is 0.5, the input feature map will first use bilinear upsampling and then use a convolution kernel with a stride of one for calculation, so (2) can be transformed into

(3) $$\begin{array}{c} y^{l}=\text{Upsample}\left(\omega_{1}*S_{1}X^{l+1}\right)+\omega_{0}*S_{1}X^{l}+\omega_{-1}*S_{2}X^{l-1}. \end{array}$$

To improve performance, integrated batch normalization (iBN) and deformable convolution networks (DCN) [33] are used in the SEPC. The calculation of iBN is based on all feature maps in the feature pyramid, rather than a single feature map, which makes the variance smaller, so that a better training effect can be achieved under a smaller batch size. DCN can maintain the scale balance between feature maps, thereby extracting features with constant scale.

In this research, we used SEPC to improve the neck network. The original neck network input consists of the output of the 3rd, 4th, and 5th CSP modules in the backbone network. To make better use of low-level features, we added the output of the second CSP module as an additional input. Then, we used two SEPC modules for feature fusion. The first SEPC module has four inputs, and the second has only three inputs. Since the DenseNet structure in the backbone network enhances the transfer of the low-level features, and considering the scale of the calculation, the additional input is only used when the first SEPC module calculates the top layer of the feature pyramid. In addition, we modified the location of DCN layer to optimize the network structure. Compared with the ordinary convolution layer, the advantage of DCN is that it can extract features with the same scale from the feature maps of different levels. However, the calculation of the DCN layer is more complicated than the ordinary convolutional layer. In the original SEPC, the DCN layer was used when calculating feature fusion. Each DCN layer will be used multiple times when calculating the feature fusion, which will bring about a substantial increase in the amount of calculation. The primary function of the SEPC module is to realize feature fusion better, and feature extraction has been completed before. Therefore, using DCN in SEPC feature fusion will only increase the amount of calculation and cannot reflect the advantages of DCN. We added DCN layers to extract features from the feature pyramid before computing the feature fusion and replaced the DCN layers in SEPC with ordinary convolutional layers. In this way, the computational complexity is reduced while retaining the advantages of DCN. Finally, Figure 7 shows our improved neck network structure.

In summary, Figure 8 shows our improved YOLOv4 model, and our main contributions are as follows. On the basis of retaining the advantages of original YOLOv4 model, we introduced the DenseNet structure to improve the performance of the backbone network, pruned the network structure to reduce the computation and keep the output dimension unchanged, and designed a new neck network to improve feature fusion effect.

## 4. Experiment and Analysis

### 4.1. Experimental Platform and Parameters

This research used Python to write the program code, and the system environment is as follows: Intel Core i9 10885H CPU, 64G RAM, Nvidia Quadro RTX 5000 Max-Q GPU, and Windows 10 operating system. All models were trained with an epoch of 300, a batch size of 16 and, an input image size of 512 × 512. The training environment is Python 3.7; the deep learning framework is PyTorch 1.8; the GPU software environment is Cuda11.0 and cudnn8.0. The initial value of the learning rate is 0.01. Cosine annealing is used as the change strategy, and the change curve of the learning rate is shown in Figure 9.

In addition, the image augmentation parameters used in the training process are shown in Table 2:

### 4.2. Evaluation Indicators of the Model

In this paper, we used precision, recall, and average precision (AP) as performance evaluation metrics. Precision is the probability of being correct in all detected targets; recall is the probability that all positive samples correctly identified; AP is the weighted mean of precision achieved at each recall value. Their calculation method is shown as follows:

(4) $$\begin{array}{c} \text{precision}=\;\frac{\text{TP}}{\text{TP}+\text{FP}},\\ \text{recall}=\frac{\text{TP}}{\text{TP}+\text{FN}},\;\\ \text{AP}=\sum_{n}\left(R_{n}\;-\;R_{n-1}\right)P_{n}, \end{array}$$

where TP is the number of positive samples that have been correctly identified; FP is the number of negative samples that have been incorrectly identified; FN is the number of positive samples that have been incorrectly identified; and *P*_*n*_ and *R*_*n*_  are the precision and recall at the nth threshold.

### 4.3. Experimental Results and Analysis

#### 4.3.1. Impact of the Improved Backbone Network

The purpose of this experiment is to verify the impact of the introduction of DenseNet structure and pruning networks on the performance of the model.  Figure 10 shows the comparative experimental results of the YOLOv4 with improved backbone network and the original YOLOv4.

Based on these measurements, the precision, recall, and AP of the model remain basically unchanged before and after modification. This means that, for the pine cone detection task, using CSPdarknet53 as the backbone network has redundancy, and the introduction of DenseNet structure or pruning the network will not affect the accuracy. However, after modifying the backbone network, the computational cost of the model dropped from 95.6 GFLOPs to 84.8 GFLOPs, an 11.3% reduction, which will increase the detection speed. In addition, Figure 11 shows the loss change process during training. After about 20 epochs, the loss value of the modified model drops faster. So, the introduction of the DenseNet structure is conducive to the feature extraction process and can make the model have better convergence effect and faster convergence speed.

#### 4.3.2. Impact of the Improved Neck Network

The purpose of this experiment is to verify the performance of the neck network designed in this paper. We trained the original YOLOv4 and the YOLOv4 with improved neck. The experimental results are shown in Figure 12.

After using the neck network we designed, the precision of the model rose from 92.8% to 94.2%; the recall rose from 83.6% to 88.1%; the AP@0.5 rose from 88.4% to 93.7%. Although precision has only a small improvement, recall and AP have significantly improved. This shows that the improved neck network can effectively enhance the effect of feature fusion. In addition, compared with the original neck network, the improved neck network removes some extra convolutional layers, so its computational complexity is smaller.

#### 4.3.3. Overall Performance Comparison

In this experiment, we tested the performance of the overall improved YOLOv4. As shown in Figure 13, the precision of our improved YOLOv4 is 96.1%, the recall is 90.1%, the AP@0.5 is 95.8%, and the AP@0.5 : 0.95 is 68.3%. For the pine cone detection task, our improved backbone network and neck network produced a coupled response. Compared with using the improved backbone network or the improved neck network alone, combining them can better improve the performance of the model. In addition, the computational cost of our improved YOLOv4 is 75.3 GFLOPs, which is 21.2% less than the original YOLOv4, but our improved model has higher accuracy. Therefore, our improvement method is effective.

Additionally, the test results of the whole picture are compared in Figure 14. When the target is blocked or the target is tiny, the original YOLOv4 has many missed and false. The effect of the improved YOLOv4 is significantly better than the unimproved method. The red mark in the figure is the test result of the same area. Through the comparison, it can be clearly seen that the improved model has detected the target that was missed by the original YOLOv4, and the improved model has a higher confidence.

#### 4.3.4. Comparison with Other Models

The existing detection models are generally designed for multiclass target detection tasks, and their detection objects include large, medium, and small targets, so they may not be effective for specific detection tasks. Our improved model is only for pine cone detection tasks, and all the improved methods are based on improving the detection accuracy of small target pine cones. In order to verify the superiority of our improved model, we compared it with RetinaNet, Faster R-CNN, YOLOv3, and original YOLOv4, and the results are shown in the Table 3. It can be seen that the AP value of our model is 12.1% higher than RetinaNet, 10.6% higher than Faster R-CNN, 10.1% higher than YOLOv3, and 7.4% higher than original YOLOv4. The detection speed of our model is 4.6 ms faster than RetinaNet, 31.2 ms faster than Faster R-CNN, 1.2 ms slower than YOLOv3, and 1.1 ms faster than original YOLOv4. Overall, our model has the highest AP value, far exceeding other models. Although the detection speed is slightly lower than the YOLOv3, it can satisfy the requirements of real-time pine cone detection.

## 5. Conclusions

This paper proposes a detection method for pine cone based on an improved YOLOv4 model. In the improved design of the network architecture, in order to make better use of the shallow feature information, we replaced the CSP module in the original YOLOv4 network with the CSPDenseNet module. To reduce the computational complexity and keep the output dimension unchanged, the backbone network was appropriately pruned. To improve the recognition accuracy of the pine cone target, we changed the feature map fusion mode in the original YOLOv4 and designed a new neck network based on SEPC.

Through manual collection and use of crawling technology, we created a pine cone data set containing 1411 images. The test results on this dataset show that the proposed improved network model can effectively identify the pine cone target in a complex background. The precision, recall, and AP of the model are 96.1%, 90.1%, and 95.8%, respectively, and the average detection speed of each image is 7.1 ms. Compared with RetinaNet, Faster R-CNN, and original YOLOv4, the AP value of the proposed improved YOLOv4 model increased by 12.1%, 10.6%, and 7.4%, respectively, and the detection time was reduced by 4.6 ms, 31.2 ms, and 1.1 ms, respectively. Although the improved model detection speed is 1.2 ms slower than YOLOv3, the accuracy is 10.1% higher than it. In general, the performance of the improved model is better than the existing model.

The method proposed in this paper can effectively detect pine cones and can provide technical references for pine cone yield estimation and automatic picking. However, it still has room for improvement. Future work will focus on collecting images of more miniature pine cones, collecting different kinds of pine cone images, and optimizing low-performance computing boards. In addition, the combination of cameras with infrared detectors, LiDAR, and the crewless aerial vehicle is also worth researching.

## Figures and Tables

**Figure 1:** Different images of pine cones in the data set. (a) Pine cones on trees; (b) pine cones on ground; (c) mature pine cones; (d) immature pine cones.

**Figure 2:** The effect of data augmentation.

**Figure 3:** The YOLOv4 model structure.

**Figure 4:** Comparison of YOLOv3 with YOLOv4. (a) YOLOv3 with FPN; (b) YOLOv4 with PAN.

**Figure 5:** The CSPDenseNet structure.

**Figure 6:** Comparison of SEPC with FPN and PAN. (a) FPN; (b) PAN; (c) SEPC.

**Figure 7:** The improved neck network.

**Figure 8:** The improved YOLOv4 model.

**Figure 9:** The change curve of learning rate.

**Figure 10:** Comparison of the YOLOv4 with improved backbone network and the original YOLOv4. (a) Precision; (b) recall; (c) AP@0.5.

**Figure 11:** Loss changes during training.

**Figure 12:** Performance verification experiment of the neck network: (a) precision; (b) recall; (c) AP@0.5.

**Figure 13:** Overall performance comparison.

**Figure 14:** Whole image test comparison. (a) The original YOLOv4; (b) the improved YOLOv4.

**Table 1:** Structure of the original backbone network and the improved backbone network.

Module	Number of layers		Number of filters		Output channels
	Original	Improved	Original	Improved	
1	Residual^∗^1	Residual^∗^1	1 × 1 Conv^∗^32	1 × 1 Conv^∗^32	64
			3 × 3 Conv^∗^64	3 × 3 Conv^∗^64	

2	Residual^∗^2	Residual^∗^2	1 × 1 Conv^∗^64	1 × 1 Conv^∗^64	64
			3 × 3 Conv^∗^64	3 × 3 Conv^∗^64	

3	Residual^∗^8	Dense^∗^4	1 × 1 Conv^∗^128	1 × 1 Conv^∗^64	128
			3 × 3 Conv^∗^128	3 × 3 Conv^∗^32	

4	Residual^∗^8	Dense^∗^4	1 × 1 Conv^∗^256	1 × 1 Conv^∗^128	256
			3 × 3 Conv^∗^256	3 × 3 Conv^∗^64	

5	Residual^∗^4	Dense^∗^4	1 × 1 Conv^∗^512	1 × 1 Conv^∗^256	512
			3 × 3 Conv^∗^512	3 × 3 Conv^∗^128	

**Table 2:** Hyperparameters.

Hsv_h	Hsv_s	Hsv_v	Translate	Scale	Fliplr	Mosaic
0.015	0.4	0.4	0.1	0.4	0.5	1.0

**Table 3:** Comparison of different models.

Model	AP@0.5 (%)	Average detection time (ms)
RetinaNet	83.7	11.7
Faster R-CNN	85.2	38.3
YOLOv3	85.7	5.9
YOLOv4	88.4	8.2
Our model	95.8	7.1

## Data Availability

The dataset can be accessed upon request to the corresponding author.
